# Sanguinarine inhibits angiotensin II-induced apoptosis in H9c2 cardiac cells via restoring reactive oxygen species-mediated decreases in the mitochondrial membrane potential

**DOI:** 10.3892/mmr.2015.3841

**Published:** 2015-05-25

**Authors:** YUAN LIU, RONG JIAO, ZHEN-GUO MA, WEI LIU, QING-QING WU, ZHENG YANG, FANG-FANG LI, YUAN YUAN, ZHOU-YAN BIAN, QI-ZHU TANG

**Affiliations:** 1 Department of Cardiology, Renmin Hospital of Wuhan University, Wuhan, Hubei 430060, P.R. China; 2 Cardiovascular Research Institute of Wuhan University, Wuhan, Hubei 430060, P.R. China; 3 Xiangyang Hospital, Hubei University of Medicine, Xiangyang, Hubei 441000, P.R. China

**Keywords:** angiotensin II, sanguinarine, oxidative, H9c2 cardiac cells, apoptosis

## Abstract

Cell apoptosis induced by Angiotensin II (Ang II) has a critical role in the development of cardiovascular diseases. The aim of the present study was to investigate whether sanguinarine (SAN), a drug which was proved to have anti-oxidant, anti-proliferative and immune enhancing effects, can abolish cell apoptosis induced by Ang II. In the present study, H9c2 cardiac cells were stimulated with 10 *µ*M Ang II with or without SAN. The level of intracellular reactive oxygen species (ROS) generation was assessed using dichlorodihydrofluorescein diacetate, and changes of the mitochondrial membrane potential (MMP) were assessed using JC-1 staining. Furthermore, mRNA expression of NOX2 was determined by reverse transcription quantitative polymerase chain reaction, and apoptosis was detected by Annexin V/propidium iodide staining and flow cytometry. The expression of B-cell lymphoma 2 (Bcl-2), Bcl-2-associated X protein (Bax) as well as cleaved (c)-caspase 3 and -9 were detected by western blot analysis, and the activity of caspase 3 and -9 was detected using an ELISA. The results of the present study showed that NOX2 expression and ROS generation induced by Ang II were inhibited by SAN, and the Ang 2-induced MMP loss was also ameliorated. Furthermore, Ang II-induced H9c2 cardiac cell apoptosis as well as c-caspase 3 and -9 levels were significantly reduced by SAN. Investigation of the possible pathway involved in the anti-apoptotic effect of SAN showed that the expression of Bcl-2 was decreased, while that of Bax was increased following stimulation with Ang II, which was reversed following treatment with SAN. In addition, Ang II enhanced the activity of caspase 9 and cleaved downstream caspases such as caspase-3, initiating the caspase cascade, while pre-treatment of H9c2 cardiac cells with SAN blocked these effects. In conclusion, the findings of the present study indicated that SAN inhibits the apoptosis of H9c2 cardiac cells induced by Ang II, most likely via restoring ROS-mediated decreases of the MMP.

## Introduction

Apoptosis is a common cause of various diseases. It is one of the factors that is able to reduce cardiac contractility and can also lead to heart failure through multiple pathways. Certain studies have indicated that cardiomyocyte apoptosis promotes the transition from compensatory cardiac hypertrophy to heart failure in response to pressure overload. (1–3).

It is well established that the renin-angiotensin-aldosterone system (RAAS) is activated in cardiovascular diseases, including hypertension (4), atherosclerosis (5), left ventricular hypertrophy (LVH) (6) and heart failure (6). Angiotensin II (AngII) is the primary active peptide hormone of the RAAS, which impairs the homeostasis between the production and elimination of reactive oxygen species (ROS) through NADPH oxidase, cause a series of cascade reactions, and finally leads to cardiomyocyte hypertrophy and apoptosis (7,8). Ang II also induces H9c2 cardiac cell hypertrophy, oxidative stress, mitochondrial dysfunction and cell apoptosis through Ang II type 1 receptor activation (9,10).

Since the mitochondrial membrane potential (MMP) has central roles in cardiomyocyte apoptosis, Ang II also induces apoptosis via the mitochondrial-dependent apoptotic pathway (11); therefore, anti-oxidant supplementation may ameliorate apoptosis induced by Ang II, which may be an effective therapeutic method for cardiovascular disease.

Sanguinarine (SAN), derived from the root of *Sanguinaria canadendid* is a benzophenanthridin alkaloid (12). As a Traditional Chinese Medicine, SAN has been proved to have significant anti-bacterial, anti-oxidant, anti-proliferative, anti-tumor and immune enhancing effects (13). Previous studies indicated that SAN accelerated cell apoptosis and inhibited cell proliferation in cancer cells (14,15). A recent study by our group demonstrated that SAN exerted a significant protective effect against pressure overload-induced cardiac remodeling via inhibition of nuclear factor-κB activation (16). However, whether SAN has protective effects against Ang II-induced H9c2 cardiac cell apoptosis has remained elusive. Therefore, the present study investigated the effect of SAN on the apoptosis, ROS generation and mitochondrial dysfunction of H9c2 cardiac cells induced by Ang II.

## Materials and methods

### Cell culture

The rat cardiomyocyte-derived cell line H9c2 was obtained from the Cell Bank of the Chinese Academy of Sciences (GNR5; Shanghai, China). Cells were cultured in 1X Dulbecco's modified Eagle's medium (DMEM) basic (C11995; Gibco-BRL, Invitrogen Life Technologies, Carlsbad, CA, USA) supplemented with 10% fetal bovine serum (FBS; 10099; Gibco-BRL) and 1% penicillin - streptomycin (PS; 1308300; Gibco-BRL) at 37°C in a humidified atmosphere containing 5% CO_2_ (18 M; Sanyo, Osaka, Japan). Upon reaching 80% confluency, cells were detached with 1 ml 0.25% trypsin-EDTA (1316929; Gibco-BRL) and passaged at a 1:2-ratio. Prior to stimulation, cells were cultured with serum-free DMEM basic (1X; supplemented with 0.05% PS) for 24 h in order to eliminate the influence of FBS and synchronize the cells.

### Cell viability assay

Cell viability was measured using a Cell Counting kit-8 (CCK-8) assay (ER612; Dojindo, Kumamoto, Japan). SAN (>98%; C_2_OH_14_NO_4_) was purchased from Shanghai Winherb Medical S&T Development Co., Ltd. (Shanghai, China). The cells were seeded into 96-well plates at a density of 1×10^5^ cells/ml and starved for 24 h prior to being exposed to different concentrations of SAN, N-acetyl-L-cysteine (NAC, 1 mmol/l; 1009005; Sigma-Aldrich, St Louis, MO, USA) and co-treatment with Ang II (A9525; Sigma-Aldrich) for 12 h. After that, 10 *µ*l CCK-8 solution was added to each well followed by incubation at 37°C for 2.5 h. The samples were read at 450 nm on a Synergy HT plate reader (Bio-Tek, Winoosky, VT, USA). The means of the optical density (OD) of the five wells were used to determine the percentage of viable cells according to the following formula: Cell viability (%) = OD (treatment group)/OD (control group) ×100%.

### ROS measurement

The level of intracellular ROS generation was assessed using the fluorescent dye dichlorodihydrofluorescein diacetate (DCFH-DA; D6883; Sigma-Aldrich). After the indicated treatments, cells were washed twice with phosphate-buffered saline (PBS; Beyotime Institute of Biotechnology, Jiangsu, China) and then incubated with serum-free DMEM basic (1X) containing 10 *µ*mol/l DCFH-DA at 37°C for 30 min. After that, cells were washed with PBS three times in order to eliminate the residual DCFH-DA. Cells from each group were analyzed by measuring the excitation and emission spectrum at 488 and 525 nm, respectively, using a Synergy HT microplate reader. Data were collected and analyzed, and the mean fluorescence intensity (FI) of five wells per group were used to determine the ROS content ratio as a percentage of the control according to the following formula: ROS levels (%) = FI (treatment group)/FI (control group) ×100%. Furthermore, fluorescence microscopy (CX 21FS1C; Olympus, Tokyo, Japan) was used to confirm the results of the microplate ROS assay. In brief, after the indicated treatments for 6 h, cells were washed twice with PBS and then incubated with serum-free DMEM basic (1X) containing 10 *µ*mol/l DCFH-DA at 37°C for 30 min. Subsequently, the cells were washed with PBS three times in order to eliminate the residual DCFH-DA; the climbing glasses of cells were collected and mounted using SlowFade Gold antifade reagent with DAPI (Invitrogen Life Technologies). The fluorescence was visualized using a fluorescence microscope coupled with an image analysis system (DP2-BSW version 1.3; Olympus).

### Measurement of the mitochondrial transmembrane potential (MMP; ΔΨm)

The change of the mitochondrial membrane potential (MMP) was assessed using the fluorescent dye 5,5′,6,6′-tetrachloro-1,1′,3,3′-tetraethylimidacarbocyanine iodide (JC-1; C2005; Beyotime Institute of Biotechnology, Shanghai, China). After the designated treatment of the cells, 100 *µ*l serum-free DMEM basic (1X) and 5 *µ*g/ml JC-1 was added to the cells, followed by incubation at 37°C for 20 min. Following two washes with PBS, the FI of JC-1 monomer was analyzed by capturing excitation and emission spectra at 485 and 530 nm, respectively, with a Synergy HT. JC-1 multimer FI was analyzed via excitation and emission spectra at 528 and 590 nm, respectively. The mean values of the five wells were used to determine the percentage of FI levels according to the following formula: FI levels (%) = FI (treatment group)/FI (control group) ×100%. In addition, cells labeled with JC-1 were observed using fluorescence microscopy. JC-1 fluorescence was measured using a single excitation wavelength (485 nm) with dual emission (shift from green at 530 nm to red at 590 nm).

### Reverse transcription quantitative polymerase chain reaction (RT-qPCR)

Total RNA was isolated from H9c2 cardiac cells using TRIzol reagent (15596-026; Invitrogen Life Technologies). Their yields and purities were spectrophotometrically estimated using the absorbance at 260 nm (A260)/A280 and A230/A260 ratios using a Nanodrop 2000c (Thermo Fisher Scientific, Waltham, MA, USA). The RNA (2 *µ*g of each sample) was reverse-transcribed into cDNA using oligo (dT) primers and the Transcriptor First Strand cDNA Synthesis kit (04896866001; Roche Diagnostics, Basel, Switzerland) according to the manufacturer's instructions. SYBR Green PCR Master Mix (04707516001; Roche Diagnostics) was then used to quantify PCR amplifications using a Light Cycler 480 instrument with designated software (version 1.5; Roche Diagnostics), the PCR conditions were as follows: Initial denaturation at 94°C for 2 min, followed by 25–35 amplification cycles consisting of denaturation at 94°C for 40 sec, annealing at 58°C for 45 sec and elongation at 72°C for 1 min. NOX2 mRNA was amplified using the following primers: Forward, 5′-TGA ATC TCA GGC CAA TCA CTTT-3′ and reverse, 5′-AAT GGT CTT GAA CTC GTT ATCCC-3′. The primers were manufactured by Sangon Biotech Co., Ltd. (Shanghai, China). The housekeeping gene GAPDH was employed to normalize gene expression values, using the following primers: Forward, 5′-GAC ATG CCG CCT GGA GAAAC-3′ and reverse, 5′-AGC CCA GGA TGC CCT TTAGT-3′.

### Flow cytometric analysis of apoptosis

Apoptosis was evaluated using an Annexin V-fluorescein isothiocyanate (FITC)/propidium iodide (PI) apoptosis kit (3300222; MultiSciences Biotech, Co., Ltd, Suzhou, China). After experimental treatment, cells were harvested, washed with cold PBS and then re-suspended in 500 *µ*l 1X binding buffer and 5 *µ*l Annexin V-FITC. Following incubation in the dark at room temperature for 15 min, 10 *µ*l PI was added. Cellular fluorescence was measured by flow cytometric analysis using a FACSCalibur flow cytometer (BD Biosciences, Franklin Lakes, NJ, USA).

### Western blot analysis

The cells were lysed in RIPA lysis buffer (Wuhan Goodbio Technology Co. Ltd., Wuhan, China) containing 50 mM Tris-Hcl, 150 mM NaCl, 1% Triton X-100, 1% sodium deoxycholate, 0.1% SDS; the cells were then scraped into 1.5-ml centrifuge tubes. The cell suspension was centrifuged at 3,362 g for 30 min at 4°C, and the protein concentration was measured using a bicinchoninic acid protein assay kit (23227; Thermo Fisher Scientific, Cambridge, MA, USA) using the Synergy HT microplate reader. The cell lysates (40 *µ*g) were fractionated by 10% SDS-PAGE (12072472; Invitrogen Life Technologies). After electrophoresis with a Gel Transfer Device (IB1001; Invitrogen Life Technologies), proteins were transferred onto a polyvinylidene difluoride membrane (Millipore, Billerica, MA, USA) and incubated with the appropriate primary antibodies, including rabbit monoclonal cleaved (c)-caspase-3 (1:1,000; cat. no. 9664; Cell Signaling Technology, Danvers, MA, USA), rabbit polyclonal c-caspase-9 (1:1,000; cat. no. 9509P; Cell Signaling Technology), rabbit polyclonal Bcl-2 (1:1,000; cat. no. 2870; Cell Signaling Technology), rabbit polyclonal Bax (1:1,000; cat. no. 2772; Cell Signaling Technology) and the membrane was incubated with diluted primary antibody in 5% w/v nonfat dry milk, 1X Tris-buffered saline, 0.1% Tween^®^ 20 at 4°C with gentle agitation, overnight. Thereafter, membranes were incubated with the secondary antibody, goat anti-rabbit immunoglobulin G (926-32211; LI-COR Biosciences, Lincoln, NE, USA), for 60 min. The blots were scanned using a two-color infrared imaging system (Odyssey; LI-COR Biosciences) to quantify protein expression. Protein expression levels were normalized to GAPDH (1:1,000; cat. no. 2118, Cell Signaling Technology).

### Caspase-3 and caspase-9 activity assay

ELISA kits were used to detect the activity of caspase-3 using the caspase-3 activity kit (C1115; Beyotime Institute of Biotechnology). Caspase-9 activity was assessed using the caspase-9 activity kit (H082; Nanjing Jiancheng Bioengineering, Nanjing, China). The two indicators were measured with the corresponding detection kit according to the manufacturer's instructions.

### Statistical analysis

Data are expressed as the mean ± standard error of the mean and analyzed using SPSS 19.0 (SPSS, Inc., Chicago, IL, USA). Comparisons between two groups were performed using an unpaired Student's t-test. Differences among groups were de termined by one-way analysis of variance followed by Student-Newman-Keuls tests. P<0.05 was considered to indicate a statistically significant difference between values.

## Results

### SAN does not affect the viability of H9c2 cardiac cells

The cytotoxicity of SAN and the ROS scavenger NAC were assessed in the presence or absence of Ang II by CCK-8 assay (Fig. 1). The viability of H9c2 cardiac cells treated with various concentrations of SAN with or without Ang II was lower than that of the control group, while cell viability remained >85% in all groups (Fig. 1A). Furthermore, the viability of the H9c2 cardiac cells in the Ang II and NAC + Ang II groups was the same as that in the control group (Fig. 1B). These results indicated that SAN and NAC exerted no cytotoxic effect on H9c2 cardiac cells.

### SAN inhibits ROS generation induced by Ang II

Previous studies showed that Ang II can generate excess intracellular ROS via stimulation of NADPH oxidase (8). In the present study, a marked increase in ROS was observed in H9c2 cardiac cells treated with Ang II, while SAN suppressed ROS generation in a dose-dependent manner (Fig. 2A). Furthermore, NAC exerted a similar ROS-decreasing effect following co-treatment with Ang II (Fig. 2B). These results were further confirmed by fluorescence microscopy, which showed that the fluorescence of DCFH-DA observed in the Ang II-treated group was effectively suppressed following treatment with SAN or NAC (Fig. 3).

### SAN inhibits NOX2 mRNA expression induced by Ang II

NOX2 is a catalytic subunit of NADPH oxidase and NOX2 NADPH oxidase has an important role in ROS generation induced by Ang II. Thus, the present study investigated whether SAN was able to affect the expression of NOX2 in H9c2 cardiac cells treated with Ang II. The results showed that Ang II significantly increased NOX2 mRNA expression in H9c2 cardiac cells in a time-dependent manner, while the most effective concentration of 0.5 *µ*M SAN significantly inhibited the elevated expression of NOX2 in a time-dependent manner (Fig. 4).

### SAN ameliorates MMP loss induced by Ang II

The stability of MMP was measured in H9c2 cardiac cells after Ang II treatment. The results revealed that the stability of MMP was significantly impaired by Ang II, as the amount of JC-1 monomers was increased and that of JC-1 multimers was decreased in the Ang II-treated group compared with that in the control group. When H9c2 cardiac cells were co-treated with SAN at various concentrations, the decreased MMP as well as the amount of JC-1 monomers and -multimers were restored to normal levels in a dose-dependent manner (Fig. 5A). In the positive control group, in analogy to the effect of SAN, NAC reversed the MMP loss induced by Ang II (Fig. 5B). These results were further confirmed using fluorescence microscopy. After the indicated treatments of H9c2 cardiac cells for 24 h, cells were stained with JC-1 and red/green image densities were measured. The green fluorescence density, indicating JC-1 monomers the red fluorescence density indicating multimers. A collapse of the MMP, was markedly increased in the Ang II group, while treatment with SAN or NAC was able to shift the green fluorescence to red fluorescence and therefore a restored MMP (Fig. 6).

### SAN attenuates Ang II-induced apoptosis

Previous studies have proved that SAN is able to regulate cell apoptosis (14). Thus, the present study investigated the anti-apoptotic effect of SAN in Ang II-treated H9c2 cardiac cells. Compared with the control group, Ang II significantly promoted cell apoptosis, as shown by the Annexin V/PI staining: The early apoptotic rate was significantly enhanced (25.3%) compared to that in the control group (1.8%), while SAN and NAC attenuated the level of apoptosis, with the early apoptotic rate decreased to 14.5 and 14.4%, respectively (Fig. 7).

### SAN ameliorates the expression of apoptosis family proteins

The lysate of cells of the experimental groups was assessed regarding the expression of c-caspase 3, c-caspase 9 and Bcl-2 family proteins. The expression of c-caspase3 and c-caspase 9 was increased in the Ang II group, while the expression of the anti-apoptotic protein Bcl-2 was significantly decreased. Furthermore, the expression levels of pro-apoptotic protein Bax were increased. These results are in line with the finding that Ang II induced H9c2 cardiac cell apoptosis. Treatment with SAN or NAC was able to significantly reduce the Ang II-induced expression of c-caspase 3 and -9 as well as Bax, and to decrease the expression of Bcl-1 (Fig. 8). The results therefore indicated that SAN is able to block apoptosis of cardiac cells by interfering with the mitochondrial-mediated apoptosis signaling pathway.

### SAN inhibits caspase-3 and caspase-9 activation induced by Ang II

Caspase-3 and caspase-9 activity were significantly increased in Ang II-treated H9c2 cardiac cells, while SAN and NAC significantly inhibited Ang II-induced caspase activation (Fig. 9). This result further confirmed the mechanism of action of SAN as an inhibitor of the mitochondrial-mediated apoptotic pathway to inhibit apoptosis of cardiac cells.

## Discussion

The present study demonstrated that Ang II increased ROS generation, initiating a signaling cascade contributing to MMP loss and resulting in an up-regulation of apoptosis of H9c2 cardiac cells. Of note, SAN ameliorated ROS generation and MMP loss in H9c2 cardiac cells induced by Ang II, and decreased caspase 3 and -9 protein expression and activity, as well as enhancing the Bcl-2/Bax ratio. In addition, the present study demonstrated that nearly all of these pro-apoptotic factors of Ang II were eliminated by NAC as a positive control treatment. These results indicated that SAN inhibits H9c2 cardiac cell apoptosis caused by Ang II, which is likely to be due to restoration of ROS-mediated decreases of the MMP (Fig. 10).

Increasing evidence suggests that Ang II treatment significantly increases NADPH oxidase activity via the Ang II receptor, type 1, and subsequently leads to ROS generation, which can cause damage to mitochondria and lipid peroxidation (17,18). A study by Chu *et al* (19) showed that Ang II was able to stimulate intracellular Ca^2+^ accumulation, which altered the MMP and caused a release of cytochrome C from the mitochondria to the cytoplasm and subsequent apoptotic cascades in neonatal rat ventricular myocytes. Chang *et al* (20) demonstrated that caspase 3 and -9 were increased in H9c2 cardiac cells stimulated by Ang II, which was confirmed by the present study. Therefore, it was hypothesized that Ang II causes mitochondrial damage and MMP loss via ROS generation and subsequent activation of apoptosis, and the present study was designed to investigate whether SAN was able to decrease ROS generation in H9c2 cardiac cells and ameliorate MMP loss and apoptosis caused by Ang II.

Numerous studies have focused on SAN as an anti-oxidant and anti-inflammatory drug (21–23). Ahmad *et al* (14) showed that low-dose SAN (1 *µ*M) treatment of A431 cells resulted in a significantly decreased cell viability and an enhanced apoptotic index, while this treatment had no effect on NHEK normal keratinocyte cells, which exclusively showed necrotic staining at the high doses of 2–5 *µ*M. In the present study, in order to avoid H9c2 cardiac cell necrosis, a maximum SAN concentration of 0.5 *µ*M was used, and after treatment for 12 h, the viability of H9c2 cardiac cells treated with different concentrations of SAN with or without Ang II was lower than that in the control group, while always remaining >85%; this indicated that SAN had no significant toxicity to H9c2 cardiac cells.

The chemical reactivity of SAN is based on the nucleophilic character of its iminium moiety, which may participate in oxidant scavenging and/or enzyme inhibition (24). SAN was shown to inhibit phorbol myristate-induced oxidative burst (25), and the most important enzyme in oxidative burst is the NADPH oxidase complex (26). SAN may have exerted its anti-oxidative function by impairing the activity of the NADPH enzyme, which is supported by a study by Qin et al (26), which demonstrated that SAN is an enzyme inhibitor rather than an ROS scavenger. NADPH oxidases are transmembrane enzymes designated to produce super-oxide by transferring an electron from NADPH to molecular oxygen. NOX2 is a major NADPH oxidase isoform expressed in cardiac cells (27,28), and it is well established that several actions of NOX2 NADPH in cardiac remodeling are activated through activation by Ang II, and alongside tumor necrosis factor alpha, it constitutes the main source of ROS generation (29,30). NOX2-derived ROS has a major role in the regulation of cardiac hypertrophy, apoptosis, fibrosis and mitochondrial dysfunction (26,31,32). As NOX2 NADPH oxidase has an important role in ROS generation induced by Ang II, it was speculated that SAN impaired the generation of ROS through decreasing the expression of NOX2 NADPH oxidase. These hypotheses were confirmed by the results of the present study, showing that SAN (0.5 *µ*M) inhibited NOX2 NADPH oxidase activity in a time-dependent manner and that ROS generation induced by Ang II was also inhibited by SAN in a dose-dependent manner.

In the present study, ROS were significantly elevated and the MMP was declined in the Ang II-treated group. A high level of ROS production may cause mitochondrial oxidative attack as well as accumulating damage to mitochondrial DNA and proteins, which further stimulates ROS generation (ROS-induced ROS release) (33). These interactions cause mutual damage and lead to H9c2 cardiac cell apoptosis, which, however, was demonstrated to be inhibited by pre-treating the H9c2 cardiac cells with SAN. NOX2 levels induced by Ang II were also inhibited by SAN, and Ang II-induced H9c2 cardiac cell apoptosis as well as c-caspase 3 and -9 expression were significantly reduced by SAN. Furthermore, the present study investigated the possible molecular pathway underlying the anti-apoptotic effect of SAN. The results showed that the expression of Bcl-2 was decreased, while Bax increased following treatment with Ang II, which was rescued by treatment with SAN. In addition, Ang II enhanced the activation of caspase 9 and caspase 3, while pre-treatment of H9c2 cardiac cells with SAN blocked these effects. Pre-treatment with NAC as a positive reference exerted similar effects to those of SAN on protein expression, changes in the MMP and the apoptotic index in response to Ang II.

In conclusion, the present study provided novel insight into the cardioprotective effect of SAN as well as the underlying molecular mechanisms. SAN inhibits ROS generation, MMP loss and apoptosis of H9c2 cardiac cells induced by Ang II, possibly via inhibiting NOX2 and the mitochondrial-mediated apoptotic pathway. Although the precise mechanism remains to be fully elucidated, the present study may contribute to the selection of SAN as a candidate drug for the treatment or prevention of cardiovascular diseases.

## Figures and Tables

**Figure 1:** Effects of SAN on cell viability of H9c2 cardiac cells. (A) Cells were treated with Ang II (10 *µ*M) and/or the specified concentrations of SAN (0.125, 0.25, 0.5 *µ*M) for 12 h; (B) Cells were treated with Ang II (10 *µ*M) and/or NAC (1 mmol/l) for 12 h. Cell viability was measured and expressed as the mean ± standard error of the mean for three independent experiments. ^*^P<0.01 vs. 0 *µ*M SAN, ^#^P<0.05 vs. 0 *µ*M SAN. SAN, sanguinarine; Ang, angiotensin; NAC, *N*-acetylcysteine.

**Figure 2:** SAN inhibited ROS generation induced by Ang II. (A) H9c2 cells were pre-cultured with SAN (0.125, 0.25 or 0.5 *µ*M) for 40 min and then incubated in the presence of SAN (0.125, 0.25 or 0.5 *µ*M) with 10 *µ*M Ang II for a further 12 h.; (B) H9c2 cells were grown with AngII (10 *µ*M) in the absence or presence of NAC (1 mM) for 12 h. ROS generation was measured and expressed as the mean ± standard error of the mean for three independent experiments. ^#^P<0.01 vs. control; ^*^P<0.01 vs. Ang II group. SAN, sanguinarine; Ang, angiotensin; ROS, reactive oxygen species; NAC, *N*-acetylcysteine.

**Figure 3:** SAN inhibits reactive oxygen species generation induced by Ang II. The climbing glasses of cells were collected and mounted using SlowFade Gold antifade reagent with DAPI. Changes in the density of dichlorodihydrofluorescein diacetate fluorescence (green) were confirmed by fluorescence microscopy (magnification, x200). (A) Control; (B) Ang II (10 *µ*M); (C) Ang II (10 *µ*M) + SAN 0.5 *µ*M; (D) Ang II (10 *µ*M) + *N*-acetylcysteine (1 mM). Ang, angiotensin; SAN, sanguinarine.

**Figure 4:** SAN inhibits NOX2 mRNA expression induced by Ang II. H9c2 cardiac cells were pre-treated with SAN (0.5 *µ*M) for 40 min and thereafter, cells were co-treated with Ang II (10 *µ*M) for the indicated durations (0, 6 and 12 h). Values are expressed as the mean ± standard error of the mean. ^#^P<0.01 vs. control group; ^*^P<0.01 vs. Ang II group at the same time-point. SAN, sanguinarine; Ang, angiotensin.

**Figure 5:** Effects of SAN on MMP loss induced by Ang II. (A) H9c2 cardiac cells were pre-treated with various concentrations (0.125, 0.25 and 0.5 *µ*M) of SAN for 40 min prior to being co-treated with Ang II (10 *µ*M) for 24 h. JC-1 staining indicated that in the Ang II group, the amount of monomers was increased, while that of multimers was decreased compared with that in the control group. When H9c2 cardiac cells were co-treated with the indicated concentrations of SAN, the decreased MMP returned to normal and (a) the number of JC-1 multimers was increased, while (b) monomers were decreased. (B) Treatment of the cells with NAC (1 mM) and Ang II (10 *µ*M) for 24 h caused similar changes in the MMP changes to that following treatment with SAN, with (a) increases in JC-1 multimers and (d) decreases in monomers. Values are expressed as the mean ± standard error of the mean for three independent experiments. ^#^P<0.01 vs. control; ^*^P<0.01 vs. Ang II group. SAN, sanguinarine; Ang, angiotensin; ROS, reactive oxygen species; NAC, *N*-acetylcysteine; MMP, mitochondrial membrane potential.

**Figure 6:** Effects of SAN on mitochondrial membrane potential loss induced by Ang II. The density of JC-1 staining was assessed by fluorescence microscopy (magnification, x200). (A) Control; (B) Ang II (10 *µ*M); (C) Ang II (10 *µ*M) + SAN 0.5 *µ*M; (D) Ang II (10 *µ*M) + *N*-acetylcysteine (1 mM). Ang, angiotensin; SAN, sanguinarine.

**Figure 7:** SAN inhibits H9c2 cardiac cell apoptosis induced by Ang II. Flow cytometry dot plots showing necrotic cells (Annexin V−/PI+) in the upper left, late apoptotic cells (Annexin V+/PI+) in the upper right, early apoptotic cells (Annexin V+/PI−) in the lower right and viable cells (Annexin V−/PI−) in the lower left. (A) Control group, the percentage of early apoptotic cells was 1.8%; (B) Stimulated by Ang II (10 *µ*M) only, the percentage of early apoptotic cells was 25.3%; (C) Stimulated by Ang II (10 *µ*M) and SAN (0.5 *µ*M), the percentage of early apoptotic cells dropped to 14.5%; (D) Stimulated by Ang II (10*µ*M) and NAC (1 mM), the percentage of early apoptotic cells dropped to 14.4%. Values are expressed as the mean ± standard error of the mean for three independent experiments. SAN, sanguinarine; Ang, angiotensin; NAC, *N*-acetylcysteine; FITC, fluorescein isothiocyanate; PI, propidium iodide.

**Figure 8:** (A and B) Effects of SAN on the protein expression of c-caspase 3 and -9 as well as Bax and Bcl-2. The protein levels of c-caspase 3 and -9 as well as Bax were increased following stimulation with Ang II (10 *µ*M) for 24 h. Levels of Bcl-2 were markedly decreased following a further 24-h-incubation with Ang II. Treatment with (Ab) SAN (0.5 *µ*M) and (Bb) NAC (1 mM), decreased the levels of c-caspase 3 and -9 as well as Bax, while markedly increasing Bcl-2 levels. Values are expressed as the mean ± standard error of the mean for three independent experiments, ^#^P<0.01 vs. control; ^*^P<0.01 vs. Ang II group. Bcl-2, B-cell lymphoma 2; Bax, Bcl-2-associated X protein; SAN, sanguinarine; Ang, angiotensin; NAC, *N*-acetylcysteine; c-caspase, cleaved caspase.

**Figure 9:** Effects of SAN on the activities of (A) caspase-3 and (B) caspase-9. After stimulation by Ang II (10 *µ*M), the activity of caspase-3 and caspase-9 was significantly increased, while the activity of caspase-3 and caspase-9 was significantly decreased after SAN (0.5 *µ*M) or NAC (1 mM) treatment. Values are expressed as the mean ± standard error of the mean for three independent experiments, ^#^P<0.01 vs. control; ^*^P<0.01 vs. Ang II group. SAN, sanguinarine; Ang, angiotensin; NAC, *N*-acetylcysteine.

**Figure 10:** Schematic showing the proposed mechanism of action of SAN. SAN inhibits Ang II-induced apoptosis in H9c2 cardiac cells via restoring ROS-mediated decreases in the MMP. SAN inhibits ROS generation and MMP loss induced by Ang II in H9c2 cells. Furthermore, caspase 3 and caspase 9 protein expression and activity were decreased and the Bcl-2/Bax ratio was enhanced accordingly. SAN, sanguinarine; Ang, angiotensin; Bcl-2, B-cell lymphoma 2; Bax, Bcl-2-associated X protein; MMP, mitochondrial membrane potential.
